The article "Identifying Active Compounds and Mechanisms of Citrus changshan-Huyou Y. B. Chang against URTIs-Associated Inflammation by Network Pharmacology in Combination with Molecular Docking" was published in 2022. Journal: Evid Based Complement Alternat Med.

# Identifying Active Compounds and Mechanisms of *Citrus changshan-Huyou* Y. B. Chang against URTIs-Associated Inflammation by Network Pharmacology in Combination with Molecular Docking

**DOI:** 10.1155/2022/2156157

**Published:** 2022-07-13

**Authors:** Shiyi Chen, Wenkang Huang, Xiaoyu Li, Lijuan Gao, Yiping Ye

**Affiliations:** School of Pharmacy, Hangzhou Medical College, Hangzhou, Zhejiang, China

## Abstract

**Purpose:**

The ripe fruits of *Citrus changshan-huyou*, known as Quzhou Fructus Aurantii (QFA), have been commonly used for respiratory diseases. The purpose of this study was to investigate their active compounds and demonstrate their mechanism in the treatment of upper respiratory tract infections (URTIs) through network pharmacology and molecular docking.

**Methods:**

The prominent compounds of QFA were acquired from TCMSP database. Their targets were retrieved from SwissTargetPrediction database, and target genes associated with URTIs were collected from DisGeNET and GeneCards databases. The target protein-protein interaction (PPI) network was constructed by using STRING database and Cytoscape. Gene Ontology (GO) and Kyoto Encyclopedia of Genes and Genomes (KEGG) were enriched. Visual compound-target-pathway network was established with Cytoscape. The effects of compounds were verified on the inhibitory activities against phosphoinositide 3-kinases (PI3Ks). Finally, the molecular docking was carried out to confirm the binding affinity of the bioactive compounds and target proteins.

**Results:**

Five important active compounds, naringenin (NAR), tangeretin (TAN), luteolin (LUT), hesperetin (HES), and auraptene (AUR), were obtained. The enrichment analysis demonstrated that the pathways associated with inflammation mainly contained PI3K/Akt signalling pathway, TNF signalling pathway, and so on. The most important targets covering inflammation-related proteins might be PI3Ks. *In vitro* assays and molecular docking exhibited that TAN, LUT, and AUR acted as PI3K*γ* inhibitors.

**Conclusion:**

The results revealed that QFA could treat URTIs through a multi-compound, multi-target, multi-pathway network, in which TAN, LUT, and AUR acted as PI3K*γ* inhibitors, probably contributing to a crucial role in treatment of URTIs.

## 1. Introduction

Upper respiratory tract infections (URTIs) include nasopharyngitis (common cold), sinusitis, pharyngitis, laryngitis, and laryngotracheitis, which is a common infection in children generally caused by viral, respiratory infection in the mouth, nose, throat, larynx (voice box), and trachea (windpipe) [1]. Complications or deaths due to virus infections are often associated with inflammation events, which cause more harm in children. For example, the seasonal influenza A virus (IVA) infects the respiratory tract, causing epithelial damage, pulmonary infiltration, hypoxemia, and even leading to acute respiratory distress syndrome (ARDS) [2]. Currently, there still a lack of antiviral drugs specifically for the treatment of URTIs, although analgesics and antipyretics are benefit for relieving symptoms such as pain and fever. Antibiotics are ineffective to treat viral infections, and inappropriate use of them for URTIs in Chinese children remains rampant [3]. Therefore, it is urgent to reduce antibacterial treatment and use symptomatic drug properly, especially for child patients [4]. Traditional Chinese medicine (TCM) was widely used for prevention and treatment of URTIs. Accumulating evidence has indicated that anti-inflammatory effect of TCM plays an important role in the treatment process, through nuclear factor kappa-B (NF-*κ*B), phosphoinositide 3-kinase (PI3K)/Akt, extracellular signal-regulated kinase (ERK), and signal transducer and activator of transcription 3 (STAT3) signalling pathways [5–7].

Quzhou Fructus Aurantii (QFA), formerly known as Changshan Huyou, the ripe fruits of *Citrus changshan-huyou* Y. B. Chang, are commonly used for respiratory diseases (such as dry cough after catching a cold) and digestive system diseases [8, 9]. According to Quzhou Prefecture Chronicles and Changshan County annals, the medicinal history of QFA can be traced back to the Qing Dynasty. With the time going, it was officially included in Zhejiang Traditional Chinese Medicine Processing Standards (2015 edition), as one of the genuine medicinal materials of new “Zhebawei” in Zhejiang Province and “Quliuwei” in Quzhou City, Zhejiang Province of China. Pharmacological research indicated that the water extract of QFA had antitussive and expectorant effects [10]. Recently it was reported that QFA extracts had anti-inflammatory effect on acute lung injury (ALI) [11] and could also prevent obesity, as well as associated metabolic diseases, such as hyperlipidemia and diabetes [12–14]. The major active components of QFA were considered to be flavonoids, alkaloids, and volatile oils. The flavonoids might be the main ingredients in treatment of URTIs which displayed anti-inflammatory effects [15, 16]. However, the specific compounds that exert these effects and their molecular mechanisms remain unclear.

With the support of the local government, the research and development of QFA are highly expected. TCM is characterized by comprehensive medical effects with complex matrices and multiple therapeutic targets. Therefore, it is difficult to elucidate the underlying molecular mechanisms. Compared with experimental research, computational biology research is an option to identify targets and signalling pathway in less time. In the present study, network pharmacology was used for evaluating molecular mechanisms by analyzing the main active compounds and targets of QFA. The inhibitory activities of main active compounds on targets were verified *in vitro*. At last, molecular docking was also applied to observing the binding affinity of ligand-target to confirm the inhibitory active compounds and targets.

## 2. Materials and Methods

### 2.1. Materials

Naringenin (PS010691, >99.0%), tangeretin (PS010637, >98.0%), luteolin (PS010346, >99.0%), hesperetin (PS000219, >98.0%), and auraptene (PS010582, >98.0%) were purchased from Chengdu Push Bio-technology Co., Ltd. (Sichuan, China). PI3K*α* (p110*α*/p85*α*) was purchased from Invitrogen (Carlsbad, California, USA). PI3K*β* (p110*β*/p85*α*) was purchased from Eurofins (Brussels, Belgium). PI3K*γ* (p120*γ*) and PI3K*δ* (p110*δ*/p85*α*) were purchased from Sigma-Aldrich (St. Louis, MO, USA). ADP-Glo Kinase Assay Kit was purchased from Promega (Madison, WI, USA). PIP2 was purchased from Life Technologies (Carlsbad, California, USA). Dimethyl sulfoxide (DMSO) and ethylenediaminetetraacetic acid disodium salt (EDTA) were purchased from Sigma-Aldrich (St. Louis, MO, USA). PI103 (Lot number: 3 A/122414), a multi-targeted PI3K inhibitor, was purchased from Tocris Bioscience (Bristol, UK).

### 2.2. Screening Compounds of QFA

The PubChem database (https://pubchem.ncbi.nlm.nih.gov/) was used for retrieving the 2D chemical structure. Traditional Chinese Medicine Systems Pharmacology Database with Analysis Platform (TCMSP, https://old.tcmsp-e.com/tcmsp.php/) provided pharmacokinetic properties for natural compounds involving oral bioavailability, drug-likeness, intestinal epithelial permeability, blood-brain barrier, and aqueous solubility. By entering the molecule name contained in QFA in the search box to search, the compounds with oral bioavailability (OB) ≥20% and drug-like components ≥0.18 were displayed. Then the active compounds were analyzed to identify biological target genes in the SwissTargetPrediction database (https://www.swisstargetprediction.ch/).

### 2.3. URTIs Target Collection and Potential Target Prediction

The DisGeNET database (https://www.disgenet.org/home/) and GeneCards database (https://www.genecards.org/) were used for collecting URTIs encoding genes with “upper respiratory tract infection,” “bronchitis,” and “pharyngitis” as keywords as described in the literature. Venny 2.1.0 (bioinfogp.cnb.csic.es/tools/venny/) was used to map drug targets of QFA to the disease targets of URTIs.

### 2.4. Protein-Protein Interaction (PPI) Network and Compound-Disease-Target Network

The potential targets were input into STRING database (https://www.string-db.org/) to obtain the targets PPI network. Cytoscape 3.7.1 was applied to constructing the PPI network and Compound-Disease-Target network. Network Analyzer, a network topology analysis plug-in in Cytoscape, was used for topological analysis of PPI networks.

### 2.5. Gene Ontology (GO) and Kyoto Encyclopedia of Genes and Genomes (KEGG) Pathway Enrichment Analyses

The potential targets were input into Metascape databases (https://metascape.org/) and selected the species as “*Homo sapiens*.” To perform GO, threshold was set to a *p* value <0.01, a minimum count of 3, and an enrichment factor >1.5 [17]. KEGG function was used for doing pathway analysis, and the top 10 KEGG pathways with a *p* value <0.01, a minimum count of 3, and an enrichment factor >1.5 were selected.

### 2.6. Construction of the Compound-Target-Pathways Network of QFA

Visual compound-target-pathway network was established with Cytoscape 3.7.1 to reflect the complex relationships. Network Analyzer was used for analyzing the network. The degree value represents the number of connections between those nodes. The size of node is related to the degree value. The larger the value is, the more interrelated the compound, target, or pathway is.

### 2.7. In Vitro Experimental Validation for Inhibition of PI3Ks

The ADP-Glo™ Kinase Assay is a luminescent kinase assay that measures ADP caused by a kinase reaction. ADP-Glo™ Kinase Assay Kit and PI3 Kinases (PI3K*α*, *β*, *γ*, and *δ*) were used for the assay. Compounds in DMSO solution and PI3 Kinases solution were diluted and transferred to assay plate by Echo (Echo liquid handler 550, Labcyte, SN: E5XX-1045). Test compounds were diluted to the highest concentration (40 *μ*M) and then diluted to the final concentrations of 20, 10, 5.0, 2.5, 1.25, and 0.625 *μ*M, respectively. 50 nL of each of them was transferred to a 384-well plate as assay plate. Kinase solutions of PI3K*α*, PI3K*β*, PI3K*γ*, and PI3K*δ* were diluted to concentrations of 0.30, 0.60, 5.00, and 2.40 *μ*g/mL (2-fold the final concentration), respectively. 2.5 *μ*L of kinase solution was added to each well of the assay plate except for control wells (2.5 *μ*L of 1 × kinase buffer was added instead). After shaking the plate, 2.5 *μ*L of substrate solution was added to each well to start reaction, and the final concentrations of PIP2 and ATP were 50 *μ*M and 25 *μ*M, respectively. The assay plate was covered and incubated at room temperature for 1 h. 5 *μ*L of ADP-Glo reagent was then added to each well to stop the reaction. Subsequently, the mixture was treated briefly with centrifuge rotor (Avanti J-15R, Beckman Coulter, SN: JBR20A055), shaken slowly, and equilibrated for 120 min. Then, 10 *μ*L kinase detection solutions was add to each well, followed by equilibration for 30 min before reading on a plate reader for luminescence. Finally, conversion data was collected on Envision (2104 Multilabel Reader, Perkin Elmer, SN: 1041048) and relative light unit (RLU) values were converted to inhibition values using the formula of (sample RLU-min)/(max-min) × 100. Herein, “min” means the RLU of no enzyme control and “max” means the RLU of DMSO control. The results were shown as graph in percentage of kinase inhibition in comparison with positive and negative control, and the IC_50_ values were calculated.

### 2.8. Molecular Docking Analysis

The 3D structure of active substance of QFA was modelled by utilizing the sketcher toolbars within SYBYL-X 2.0 software. The receptor was searched from the RCSB PDB database (https://www.rcsb.org/). The docking calculations were performed by the Flex Dock program within SYBYL-X 2.0. PyMOL software (the PyMOL Molecular Graphics System, Version 2.0, Schrodinger, LLC.) was used for performing ligand/receptor analysis.

## 3. Results

### 3.1. Compounds in QFA Associated with Biological Targets

According to the oral bioavailability (OB) and drug-likeness (DL) criteria, six compounds were retrieved: naringenin (NAR), tangeretin (TAN), luteolin (LUT), nobiletin (NOB), hesperetin (HES), and auraptene (AUR) (Table 1). Based on six compounds, Caco-2 permeability and drug half-life data were collected to determine pharmacokinetics of QFA compounds. The results indicated that AUR had the highest Caco-2 permeability and NAR had the longest drug half-life.

Six compounds corresponded to 92, 103, 103, 9, 103, and 113 targets from the SwissTargetPrediction database, respectively. After removing the duplicated genes, a total of 287 targets were finally retrieved from the SwissTargetPrediction database.

### 3.2. Predicting Target Proteins for URTIs

1951 possible treatment targets were retrieved after removing duplicated targets from DisGeNET and GeneCards database. Further, by Venny 2.1 drawing software, the 287 druggable targets were mapped to 1951 URTIs-related disease targets. Finally, 117 target proteins of corresponding active compounds of QFA were identified to be potential targets in treatment of URTIs. Compound-Disease-Target network is shown in Figure 1.

### 3.3. PPI Network

The 117 hub genes were further analyzed on the STRING online data platform and network establishment, and then the data was input into Cytoscape 3.7.1 to obtain the PPI network (Figure 2), which contained 113 nodes and 627 edges. The average node degree was 11.9 after analysis, and the median node degree was 9. Each circular node represented a protein target in the network. The degree value was represented by the number of lines connected to the same node, which means the importance of each node in the network. The larger the node in the PPI network is, the greater its degree value is. Each edge represented the interaction between proteins in the PPI network. The more lines there are in the PPI, the closer associations are found in the drug and the disease. There were 19 target proteins whose degree value is more than twice the median value (Figure 2, right). The degrees of AKT1, ESR1, SRC, EGFR, PTGS2, and MMP9 (58, 43, 43, 40, 38, and 33, respectively) were significantly higher than those of the other targets, suggesting that these six targets were the most important targets for the treatment of URTIs.

### 3.4. GO and KEGG Pathway Enrichment Analyses

GO terms were selected according to the *p* value parameter (*p* ≤ 0.01). Among them, a total of 1797 GO Biological Processes (BP), 92 GO Cellular Components (CC), and 140 GO Molecular Functions (MF) were enriched. The top 10 terms, which are remarkably enriched, are shown in Figures 3(a)–3(c). In terms of enrichment results of BP, the targets of QFA in the treatment of URTIs were mainly involved in the positive regulation of MAPK cascade, positive regulation of kinase activity, and protein autophosphorylation. From the enrichment results of MF, it was mainly related to protein kinase activity, phosphotransferase activity, and protein domain specific binding. According to the enrichment results of CC, transferase complex, transferring phosphorus-containing groups, protein kinase complex, and receptor complex were mainly involved.

To investigate integral regulation of URTIs-associated inflammation by QFA, a total of 299 pathways were obtained from database. The top 10 channels are displayed in Figure 3(d). The main process associated with inflammation included PI3K/Akt, tumour necrosis factor (TNF), and NF-*κ*B signalling pathways.

### 3.5. Compound-Target-Pathway Network

The compound-target-pathway network was performed by Cytoscape3.7.1 software, which contained 88 nodes (6 compound nodes, 72 targets, and 10 pathways) and 325 edges in total (Figure 4). It showed that each active compound could act on multiple targets and pathways. Based on the degree of compound-target-pathway network, five compounds, TAN, LUT, HES, NAR, and AUR, with the degree values of 36, 33, 32, 24, and 18, respectively, had larger nodes, indicating that they were probably the main active ingredients. However, the degree value of NOB was only 2. MET, MDM2, PIK3CA, IGF1R, and MMP9 were the top 5 targets, with the degree values of 9, 8, 8, 8, and 8, respectively. PI3K/Akt signalling pathway associated with inflammation had the largest nodes, indicating that it was probably the most important pathway in the treatment of URTIs with QFA. The active compounds of QFA might target at PI3Ks.

### 3.6. Inhibitory Activities of PI3K*α*, *β*, *γ*, and *δ*

Experimental effect of five main active compounds on PI3K/Akt signalling pathway has been verified by assaying their inhibition of PI3Ks *in vitro*. The IC_50_ values of five compounds towards Class I *α*, *β*, *δ*, and *γ* isoforms of human PI3 kinases were determined in the range of 0.625 to 40 *μ*M by using Promega ADP-Glo Kinase Assay Kit. As shown in Table 2, five compounds have quite different effects on PI3K*α*, *β*, *δ*, and *γ* isoforms. HES and NAR had no inhibitory activities with IC_50_ value > 40 *μ*M against PI3K*α*, *β*, *δ*, and *γ* isoforms. LUT displayed concentration-dependently inhibitory activities against PI3Ks with IC_50_ 2.49 *μ*M for PI3K*α*, 2.95 *μ*M for PI3K*β*, 5.79 *μ*M for PI3K*γ*, and 1.55 *μ*M for PI3K*δ* (Table 2 and Figure 5). However, AUR and TAN exhibited concentration-dependently isoform-selective inhibitory activities with IC_50_ 13.75 and 17.72 *μ*M against PI3K*γ*, respectively, but no inhibitory activities with IC_50_ value >40 *μ*M against PI3K*α*, *β*, and *δ* isoforms (Table 2 and Figure 5). To our knowledge, it is the first time that AUR and TAN have been reported as PI3K inhibitors.

As a potent PI3Ks inhibitor, the positive PI103 demonstrated excellent inhibition of PI3Ks with IC_50_ 7.10 nM for PI3K*α*, 13.50 nM for PI3K*β*, 85.50 nM for PI3K*γ*, and 12.50 nM for PI3K*δ* as expected.

### 3.7. Molecular Docking Analysis

The docking results are depicted in Figure 6. As shown in Figure 6(a), LUT bonded to PI3K*γ* (PDB ID: 1E8W) through six hydrogen bonds, in which the oxygen atom at the pyran (position 4; Figure 7(a)) formed hydrogen bonds with the residue TYR-867 and VAL-882, respectively. The hydroxyl at the benzene ring (position 5; Figure 7(a)) offered hydrogen bonds with the residue VAL-882. The hydroxyl at the benzene ring (position 3; Figure 7(a)) formed hydrogen bonds with the backbone O and the backbone NH of the residue LYS-833. The hydroxyl at the benzene ring (position 4; Figure 7(a)) also formed hydrogen bonds with the residues LYS-833 and ASP-841. In the docking result of TAN with PI3K*γ* (Figure 6(b)), the carbonyl group at the pyran (position 4; Figure 7(b)) bonded with the residue VAL-882. The methoxy group at the benzene ring (position 4; Figure 7(b)) formed hydrogen bonds with the residue TYR-867. By the analysis of the binding mode of AUR with PI3K*γ* (Figure 6(c)), the carbonyl group at the pyran (position 2; Figure 7(c)) formed hydrogen bond interaction to the residues GLU-880 and VAL-882. The high inhibitory activity of LUT, AUR, and TAN against PI3K*γ* would be due to these hydrogen bond interactions.

## 4. Discussion

Databases, like TCMSP database containing pharmacokinetic properties for natural compounds [18], drug genes prediction database like SwissTargetPrediction database [19], gene-related databases like DisGeNET [20] and GeneCards [21], and interaction databases like STRING, have been widely used for gathering information for network pharmacology. Besides, appropriate tools like Venny and Cytoscape were adopted. Through compound-target-pathway network, we can directly identify active compounds, targets, and pathways and understand the mechanisms between them in URTIs-associated inflammation. In this study, TAN, LUT, HES, NAR, and AUR were predicted to be the main active compounds related to URTIs-associated inflammation, and MET, MDM2, PIK3CA, IGF1R, and MMP9 were the main URTIs-associated targets. In addition, the KEGG enrichment analysis proved that the PI3K/Akt signalling pathway was the most related pathway. We know that PIK3CA codes PI3Ks, inferring that the active compounds might target at PI3Ks. *In vitro* PI3Ks inhibition assay demonstrated that the compounds LUT, TAN, and AUR exhibited effective inhibition on PI3Ks. Among them, LUT displayed concentration-dependently inhibitory activities against PI3Ks including Class I *α*, *β*, *δ*, and *γ* isoforms, and AUR and TAN showed concentration-dependently isoform-selective inhibitory activities against PI3K*γ*, which were confirmed by molecular docking with tight docking of these compounds to the PI3K*γ* in several hydrogen bond interactions.

PI3Ks are the negative regulators involved in regulating anti-inflammatory responses, immune response, neurodegenerative diseases, cardiovascular diseases, and tumor [22]. Among three families of PI3Ks, Class I PI3K isoforms (PI3K*α*, *β*, *γ*, and *δ*) are the most intensively studied compared with the Class II PI3K isoforms (PI3KC2*α*, C2*β*, and C2*γ*) and a single Class III PI3K, which consists of a p85 regulatory subunit and a p110 catalytic subunit coded by PIK3CA. Class I PI3K isoforms can be further classified into Class IA isoforms PI3K*α*, *β*, and *δ* (p110*α*, p110*β*, and p110*δ*) and Class IB isoform PI3K*γ* (p110*γ*) according to different activating models [23]. As we know, Class IA isoforms PI3K*α* and *β* are ubiquitously expressed, and PI3K*γ* is expressed in granulocytes, monocytes, and macrophages, whereas the PI3K*δ* isoform is found in B- and T-cells.

Class IA PI3K isoforms are particularly implicated in human cancers [24]. Class IB isoform PI3K*γ* is expressed at very low levels under physiological conditions, while it is significantly upregulated after stress. After stress in pathological state, PI3K*γ* is constitutively enriched in leukocytes. In the airways, PI3K*γ* behaves as a trigger or a target in a plethora of respiratory diseases, especially in airway inflammation including ALI, pulmonary fibrosis, asthma, and cystic fibrosis [25]. PI3K*γ* knockout in mouse models of respiratory diseases led to strengthening immunological function and improving airway inflammation, suggesting that PI3K*γ* is a therapeutic target in inflammatory-driven respiratory diseases. Multiple lines of evidence demonstrated that inhibition of PI3K*γ* activity attenuated ventilator-induced lung damage, idiopathic pulmonary fibrosis, and asthma [26,27]. In short, PI3K*γ* has been proved to play a pivotal role in respiratory tract inflammation.

Among the active compounds from QFA, LUT has been described as an anticancer agent, as well as a potent antioxidant and a neuroprotective agent [28], which was used for treatment of lower respiratory infection [29]. PI3Ks assay results demonstrated that LUT acted as a pan-PI3K inhibitor with IC_50_ 2.49 *μ*M for PI3K*α*, 2.95 *μ*M for PI3K*β*, 5.79 *μ*M for PI3K*γ*, and 1.55 *μ*M for PI3K*δ*. It is the first time that LUT has been reported as a pan-PI3K inhibitor at kinase level. PI3Ks were considered to be the molecular target for the antimetastatic effect of LUT, because LUT can directly inhibit PI3K activities and subsequently attenuate phosphorylation of Akt [30]. Moreover, LUT had beneficial effects against lipopolysaccharide- (LPS-) induced ALI, which involved the blockade of MEK/ERK-related and PI3K/Akt-related pathways in neutrophils [31].

TAN, a flavonoid derived from citrus, has been demonstrated to exhibit neuroprotective, antidiabetic, antioxidant, and anti-inflammatory effects [32–34]. According to PI3Ks assay results, TAN was a PI3K*γ*-selective inhibitor, which might be a therapeutic drug to treat URTIs. Other studies reported that TAN could impede human respiratory syncytial virus infections and inflammation [35] and have protective effects against ovalbumin-provoked allergic respiratory asthma in Swiss albino mice [36]. Moreover, there is evidence demonstrated that TAN had antiasthmatic effects partly via regulating PI3K signalling pathway [37].

AUR, a dietary coumarin in citrus fruits, has been found to exert valuable pharmacological properties as anticancer, antibacterial, antiprotozoal, antifungal, anti-inflammatory, and antioxidant agent [38, 39]. Furthermore, *in vitro* inhibition of PI3Ks showed that AUR was a PI3K*γ*-selective inhibitor which exhibited stronger activity than TAN, suggesting that AUR has a therapeutic effect on URTIs-associated inflammation. Other studies had confirmed that AUR suppressed inflammatory responses in activated RAW 264 macrophages [40, 41]. It was also reported that AUR could treat Th2 cells diseases such as asthma by inhibiting cell proliferation, decreasing the levels of cytokines (IL-4, IL-10, and IFN-*γ*) and NF-*κ*B, and reducing nitric oxide (NO) production in phytohemagglutinin (PHA) stimulation [42].

According to the KEGG enrichment analysis, TNF signalling pathway was also the related pathway involved in URTIs-associated inflammation. TNF is a key proinflammatory cytokine and has been implicated in many inflammatory lung pathophysiology, including asthma, chronic bronchitis, chronic obstructive pulmonary diseases (COPD), ALI, and ARDS [43]. Several lines of evidence showed that TNF-*α* level was upregulated in asthmatic patients [44, 45]. From the enrichment results of BP, positive regulation of protein serine/threonine kinase (RIPK) had been enriched, which is a kinase that mediates necroptosis in inflammation. RIPK1, a downstream target of the TNF signalling pathway, acts as a molecular switch that induces inflammation and cell survival [46]. When the body is stressed, RIPK1 recruited to TNFR1, and a series of ubiquitination events would activate different signalling pathways [47]. Our study suggested that QFA may also be able to treat URTIs-associated inflammation by interfering with the TNF signalling pathway.

In addition to the above two signalling pathways, NF-*κ*B signalling pathway was also involved in URTIs-associated infection. NF-*κ*B is a primary transcription factor which presents in the cytoplasm with no transcriptional activity in the resting state. After stimulation, phosphorylation of I*κ*B by I*κ*B kinase results in nuclear translocation of NF-*κ*B, which regulates immune, inflammatory, cell proliferation, and apoptosis responses [48]. Li et al. found that QFA extracts attenuated the production of IL-6, IL-1*β*, and TNF-*α* in LPS-induced RAW 264.7 cells by inhibiting the NF-*κ*B signalling pathway [11]. On the basis of compound-target-pathway network and the KEGG enrichment analysis, the therapeutic effect of QFA on URTIs is related to the inhibition of NF-*κ*B signalling pathways.

## 5. Conclusions

By using the method of network pharmacological analyses, five main active compounds (NAR, TAN, LUT, HES, and AUR) of QFA were found to act on many target proteins of URTIs, which reflected the characteristics of multi-compound, multi-target, and multi-action pathways of TCM. The inflammation-related proteins like AKT and PI3Ks played a dominant role in the PPI network and in the compound-target-pathway network, suggesting that the mechanism of QFA for the treatment of URTIs was closely related to PI3K/Akt signalling pathway. The result of *in vitro* assays and molecular docking results confirmed that TAN, LUT, and AUR, as PI3K*γ* inhibitors, played a crucial role in respiratory tract inflammation. This paper preliminarily released the material basis and mechanism of QFA in treating URTIs and provided some guidance for the further research on the treatment of URTIs.

## Figures and Tables

**Figure 1:** Compound-Disease-Target network.

**Figure 2:** PPI network of QFA and URTIs intersection targets. *Left*: analysis of the 117 hub genes in the network of the anti-URTIs effects of the compounds in QFA by STRING. The red colours and big size represent the importance in the network. *Right*: analysis of the top 16 hub genes in the network with degree centrality (DC) > 18.

**Figure 3:** GO and KEGG pathway enrichment analyses of intersection target of QFA. (a) Biological Processes. (b) Molecular Functions. (c) Cellular Components. (d) KEGG pathway.

**Figure 4:** Compound-target-pathway network of QFA. The larger nodes represent more important hub nodes. The layout follows the attribute circle with the degree value, and the targets in the outer ring represent more important targets (degree value > median).

**Figure 5:** Concentration-response curves for LUT, AUR, and TAN in inhibition of PI3Ks. Promega ADP-Glo Kinase Assay Kit was used for determining inhibitory activities for Class I *α*, *β*, *δ*, and *γ* isoforms of human PI3 kinases in the range of 0.625 to 40 *μ*M. *n* = 3.

**Figure 6:** Molecular docking of LUT (a), TAN (b), and AUR (c) with receptor protein PI3K*γ*. The hydrogen bonds are shown by dashed lines.

**Figure 7:** The structures of PI3K*γ* inhibitors in QFA.

**Table 1:** Active compounds screening.

Active compounds						
Mol	NAR	TAN	LUT	NOB	HES	AUR
ID	MOL004328	MOL005814	MOL000006	MOL005828	MOL002341	MOL013434
MW	272.27	372.40	286.25	402.43	302.3	298.41
OB (%)	59.29	21.38	36.16	61.67	70.31	25.62
Caco-2	0.28	1.23	0.19	1.05	0.37	1.24
DL	0.21	0.43	0.25	0.52	0.27	0.24
HL	16.98	—	15.94	16.20	15.78	—

MW: molecular weight, OB: oral bioavailability, Caco-2: Caco-2 permeability, DL: drug-likeness, HL: drug half-life, NAR: naringenin, TAN: tangeretin, LUT: luteolin, NOB: nobiletin, HES: hesperetin, and AUR: auraptene.

**Table 2:** Compounds on inhibitory activities of PI3Ks.

Compounds	IC_50_ (*μ*M)^*∗*^			
	PI3K*α*	PI3K*β*	PI3K*γ*	PI3K*δ*
TAN	>40	>40	17.72 ± 1.16	>40
LUT	2.49 ± 0.34	2.95 ± 0.19	5.79 ± 0.10	1.55 ± 0.15
HES	>40	>40	>40	>40
NAR	>40	>40	>40	>40
AUR	>40	>40	13.75 ± 1.31	>40
PI103 (nM)	7.10 ± 0.14	13.50 ± 0.60	85.50 ± 1.88	12.50 ± 2.07

^*∗*^Values are means of three independent experiments.

## Data Availability

The data used to support the findings of this study are available from the corresponding author upon request.
